The article "Lag Synchronization of Noisy and Nonnoisy Multiple Neurobiological Coupled FitzHugh–Nagumo Networks with and without Delayed Coupling" was published in 2022. Journal: Comput Intell Neurosci.

# Lag Synchronization of Noisy and Nonnoisy Multiple Neurobiological Coupled FitzHugh–Nagumo Networks with and without Delayed Coupling

**DOI:** 10.1155/2022/5644875

**Published:** 2022-06-02

**Authors:** Malik Muhammad Ibrahim, Shazia Iram, Muhammad Ahmad Kamran, Malik Muhammad Naeem Mannan, Muhammad Umair Ali, Il Hyo Jung, Sangil Kim

**Affiliations:** ^1^Department of Mathematics, Pusan National University, Busan 46241, Republic of Korea; ^2^Department of Mathematics, Air University, Islamabad 44000, Pakistan; ^3^Department of Cogno-Mechatronics, Pusan National University, Busan 46241, Republic of Korea; ^4^School of Health Sciences and Social Work, Griffith University, Gold Coast, Australia; ^5^Griffith Center of Biomedical and Rehabilitation Engineering (GCORE), Griffith University, Gold Coast, Australia; ^6^Department of Unmanned Vehicle Engineering, Sejong University, Seoul 05006, Republic of Korea

## Abstract

This paper presents a methodology for synchronizing noisy and nonnoisy multiple coupled neurobiological FitzHugh–Nagumo (FHN) drive and slave neural networks with and without delayed coupling, under external electrical stimulation (EES), external disturbance, and variable parameters for each state of both FHN networks. Each network of neurons was configured by considering all aspects of real neurons communications in the brain, i.e., synapse and gap junctions. Novel adaptive control laws were developed and proposed that guarantee the synchronization of FHN neural networks in different configurations. The Lyapunov stability theory was utilized to analytically derive the sufficient conditions that ensure the synchronization of the FHN networks. The effectiveness and robustness of the proposed control laws were shown through different numerical simulations.

## 1. Introduction

Generally, synchronization emerges when two or more dynamical systems have strong enough coupling strength [1–3]. In 1990, Pecora and Carroll presented a pioneer study to understand the mechanism of synchronization by considering neuronal activities as chaotic systems [4]. The synchronization phenomenon has fascinated, attracted, and motivated researchers to investigate and explore the functionality of the biologically complex brain and to understand the synchronized neural firing [5]. Neuronal firing and bursting with synchronization are essential for healthy brain activities, such as decision making, executing commands, and sending/receiving information by neurons [5–7].

Over the last few decades, several researchers have studied various synchronization schemes and methodologies for chaotic systems [8–14]. Among these, lag synchronization, defined as the drive and response system that can achieve synchronization with a positive constant time lag, is a fascinating phenomenon and has been observed in electronic circuits, neuronal communications, and lasers [13, 15–20]. In many real-life scenarios, it is required to synchronize the response system at a lag with the drive system rather than at the same time owing to the limited transmission speed of signals [21–24]. For instance, in a cellular communication system, the voice from the transmitter side at time t is heard at t+*τ* time at the receiver side [21, 23]. Therefore, how to efficiently make two chaotic systems achieve lag synchronization is a critical topic that requires comprehensive investigation. Furthermore, time delays are observed in most biological systems. Due to the existence of synaptic gaps, delay plays a key role in the synchronous operation of coupled neurons [25]. The finite transmission speed of the membrane potential along the neurons' axons and time gaps due to synaptic (information transmission) and dendritic (reception) processes between neurons produce time delays in neuronal communications [26]. It is previously shown that the unmyelinated axons can cause a reduction in the transmission speed of the neurons that could result in significantly high time delays (as high as 80 m/s) in communications between neuronal networks [27, 28]. Thus, it is essential to include these time delays in mathematical modeling and analysis to better understand the communication dynamics of neurons and their networks [29, 30]. Previous studies have also shown that many factors including coupling delays, connection configuration, and noise can affect the firing dynamics of neurons. For instance, a recent study uncovered that synchronized neuronal firing could be influenced by the coupling delays present in the chemical or electrical synaptic connections [31, 32]. Furthermore, many previous studies have used neuroimaging systems to show that different brain networks are functionally connected, and they may have single or multiple couplings, i.e., a neuronal network may have connections with one or more other neuronal networks [13, 26, 33–38]. On the other hand, a single neuron has multiple axon terminals and dendrites that allow single or multiple connections with other neurons [39].

The article "Lag Synchronization of Noisy and Nonnoisy Multiple Neurobiological Coupled FitzHugh–Nagumo Networks with and without Delayed Coupling" was published in 2022. Journal: Comput Intell Neurosci.

Taking into account, numerous efforts have been made in recent years to study the lag synchronization of delayed neural networks and chaotic systems [13, 19, 21–24, 40–44]. For example, the authors of [19] investigated the lag synchronization control for memristor-based delayed coupled neuronal networks with mismatched parameters. In [23], periodically intermittent control was used to study the effect of parameter mismatch on lag synchronization of coupled delayed systems. In [21], periodically intermittent control was utilized to explore the exponential lag synchronization for neural networks with mixed delays. In [44], adaptive control was designed to investigate the lag synchronization for competitive neural networks with mixed delays and uncertain hybrid perturbations. In [43], the adaptive lag synchronization of Cohen–Grossberg neural networks with discrete delays was discussed. In addition, several researchers have utilized neuronal models without and with time delays incorporated in gap junctions to analyze and understand the lag synchronization in neurons. [5, 13, 22, 26, 31, 34, 37, 45–53] Among different models, the FitzHugh–Nagumo (FHN) neuronal model under the effect of external electrical stimulation (EES) was a favorable choice due to its medium complexity and a very close approximation of real neuronal systems. For instance, our recent study investigated and developed control schemes that guarantee the lag synchronization of unidirectional and bidirectional time-delayed ring-structured FHN neuronal systems in the presence and absence of noise [13]. Bin Zhen et al. considered two coupled FHN neurons and developed a variation of energy algorithm under the condition of no delay in time for communication to resolve the synchronization of neurons [54]. In another study, Mao et al. presented the analysis of the synchronization of two time-delayed FHN neurons to understand the root causes behind the evolution patrons and complex characteristics in neurobiological systems [55]. Muhammad Siddique et al. presented an adaptive approach by utilizing the Lyapunov Krasovskii functional to investigate the synchronization in a bounded variable time-delayed system with external disturbances [49].

In past research, researchers have investigated the interaction between neurons and their networks in different brain regions using techniques like neuroimaging systems [56–59] and used computational models to predict the complex dynamics of neurons [60, 61] and showed that noise plays an important role in the dynamical functionality of the neurons and their networks [62, 63]. The fundamentals of the noise and delay in the communication of neuronal networks are still ubiquitous but they have a very strong implication for the functionality of neurons and their networks and in general, the synchronized functionality of the brain [64, 65]. The noise has a tremendous effect as amplification of the weak neuronal signal and therefore enhances the detection of useful information in the signal [64]. The addition of noise in such networks/systems has unveiled hidden facts such as the development of the stochastic methodology to understand respective resonance [66], noise sustained synchronization [67], vibrational resonance [68, 69], chaotic resonance [70], and coherent-resonance [71] in nonlinear dynamical systems. The presence of noise in neuronal networks enforces the neurons to optimize their firing patterns which are essentially required for communications [72]. It is therefore concluded that the addition of noise in the neuronal network under time-delayed characteristics will create a more realistic picture with the cost of complexity. This also results in a challenging investigation of the synchronization process considering the drive and salve networks.

The article "Lag Synchronization of Noisy and Nonnoisy Multiple Neurobiological Coupled FitzHugh–Nagumo Networks with and without Delayed Coupling" was published in 2022. Journal: Comput Intell Neurosci.

In the light of the above, this paper presents a methodology for lag synchronization of noisy and nonnoisy multiple coupled neurobiological FitzHugh–Nagumo (FHN) master and slave networks with and without delayed coupling, under EES, external disturbances, and different parameters for each state of the networks. Each drive and slave network contains *n* coupled neurons and all neurons in both networks are connected with other neurons of the same network via synapse and there is a special junction to communicate with target cells. The interactions between neurobiological coupled neurons, namely, the coupling junctions, have a great impact on the dynamical properties of the neurobiological network. Therefore, such configuration shows more challenging and intriguing dynamical characteristics and more intricate dynamical behavior than two, three, or *n* neurons within the same network. Various novel and diverse control schemes are proposed for both multiple coupled neurobiological networks under different scenarios. These scenarios may conclude neuronal networks with and without time delays for both drive and slave networks in addition to the absence/presence of noise. Using the theory of the Lyapunov stability, we derived the necessary and sufficient conditions that ensure the synchronization of both multiple with and without delay coupled FHN neurobiological networks. Furthermore, the proposed diverse control laws have been verified by using five neurons of each network in both neurobiological networks of coupled FHN neurons under the conditions of (with/without) external noises through numerical simulations.  Figure 1 shows the general configuration of FHN networks.

The rest of the article is organized as follows. The model formulation of noisy and nonnoisy FHN multiple neurobiological networks and designing of adaptive controllers are briefly described in Section 2. In Section 3, numerical results are presented. The conclusions have been summarized in the last section.

The article "Lag Synchronization of Noisy and Nonnoisy Multiple Neurobiological Coupled FitzHugh–Nagumo Networks with and without Delayed Coupling" was published in 2022. Journal: Comput Intell Neurosci.

## 2. Model Formulation of Noisy and Nonnoisy FHN Multiple Neurobiological Networks

This section describes the formulation of the synchronization problem for two multiple neurobiological noisy and nonnoisy FHN networks with and without delay in gap junctions under EES. Different parameters for each state of both FHN networks are considered. Consequently, four different multiple neurobiological networks with nonnoisy and noisy FHN neurons are formulated and utilized for the exploration of synchronization phenomena in coupled neural networks. Each network formulated in each case consists of *n* neurons.

### 2.1. FHN Multiple without Delay Neurobiological Networks

In this section, multiple neuronal models are mathematically expressed without introducing a delay in the gap junctions dynamics, but noisy and nonnoisy networks are considered.

#### 2.1.1. Multiple without Delay Neurobiological Nonnoisy FHN Networks

Let us consider nonnoisy multiple FHN neurobiological nondelayed networks each composed of *n* neurons. Mathematically,

(1) $$\begin{array}{c} {\dot{x}}_{i1}=x_{i1}\left(x_{i1}-1\right)\left(1-r_{i1}x_{i1}\right)-x_{i2}+\sum_{j=1}^{n}g_{ij}x_{j1}+I_{i1}+d_{i1}+u_{x_{i1}},\\ {\dot{x}}_{i2}=b_{i1}x_{i1}-c_{i1}x_{i2}\;i=1,2,3,\ldots ,n, \end{array}$$

(2) $$\begin{array}{c} {\dot{y}}_{i1}=y_{i1}\left(y_{i1}-1\right)\left(1-r_{i1}y_{i1}\right)-y_{i2}+\sum_{j=1}^{n}g_{ij}y_{j1}+I_{i1}+d_{i1}+u_{y_{i1}},\\ {\dot{y}}_{i2}=b_{i1}y_{i1}-c_{i1}y_{i2}, \end{array}$$

where *x*_*i*1_, ∈*ℜ* represents membrane-potential and *x*_*i*2_ ∈ *ℜ* the recovery-variable of the *ith* neuron of neurobiological FHN drive network, respectively, where *y*_*i*1_ ∈ *ℜ* represents membrane-potential and *y*_*i*2_ ∈ *ℜ* the recovery-variable of the *i*^th^ neuron of neurobiological FHN slave network, respectively, *r*_*i*1_, *b*_*i*1_, and *c*_*i*1_ are positive parameters, *I*_*i*1_=(Α/*ω*)cos(*ωt*) is the EES with frequency *ω* and *A* amplitude, *d*_*i*1_ is the ionic gate disturbance, *u*_*x*_*i*1__ and *u*_*y*_*i*1__ is the *i*^th^ control parameter of the drive and slave networks respectively, and *G*=(*g*_*ij*_)_*N*×*N*_ representing the topology of the network and is known as coupling matrix whose elements are defined as below:

(3) gij=gij≥0,if i↔j,∀i≠j,gij=0,if i↔j,∀i≠j,gij=−∑j=1j≠iNgij∀i≠j.

In addition, we assumed that *I*_11_=*I*_21_=⋯=*I*_*n*1_.

#### 2.1.2. Multiple without Delay Neurobiological Noisy FHN Networks

Let us consider noisy multiple FHN neurobiological nondelayed networks composed of n neurons. Mathematically,

(4) $$\begin{array}{c} {\dot{x}}_{i1}=x_{i1}\left(x_{i1}-1\right)\left(1-r_{i1}x_{i1}\right)-x_{i2}+\sum_{j=1}^{n}g_{ij}x_{j1}+I_{i1}+d_{i1}+\xi_{i1},\\ {\dot{x}}_{i2}=b_{i1}x_{i1}-c_{i1}x_{i2}\;i=1,2,3,\ldots ,n, \end{array}$$

(5) $$\begin{array}{c} {\dot{y}}_{i1}=y_{i1}\left(y_{i1}-1\right)\left(1-r_{i1}y_{i1}\right)-y_{i2}+\sum_{j=1}^{n}g_{ij}y_{j1}+I_{i1}+d_{i1}+\xi_{i1}+u_{y_{i1}},\\ {\dot{y}}_{i2}=b_{i1}y_{i1}-c_{i1}y_{i2}, \end{array}$$

where *ξ*_*i*1_ is the Gaussian noise [13] sources having zero mean and correlation function:

(6) $$\begin{array}{c} \langle \xi_{i1}\left(t\right)\xi_{i1}\left(t^{\prime }\right)\rangle =2\;D\delta \left(t-t^{\prime }\right). \end{array}$$

The article "Lag Synchronization of Noisy and Nonnoisy Multiple Neurobiological Coupled FitzHugh–Nagumo Networks with and without Delayed Coupling" was published in 2022. Journal: Comput Intell Neurosci.

#### 2.1.3. Nonlinear Control Design for Multiple without Delay Neurobiological FHN Networks

The error states of the neurobiological FHN systems formulated in equations (1) and (2) and (4) and (5) can be designed as follows:

(7) $$\begin{array}{c} e_{x_{i1}}=\frac{x_{i1}-y_{i1}}{2},\\ e_{y_{i1}}=\frac{x_{i2}-y_{i2}}{2}. \end{array}$$

Taking the derivative of the error system (7) with respect to time, we can obtain

(8) $$\begin{array}{c} \left[\begin{array}{c} {\dot{e}}_{x_{11}}\\ {\dot{e}}_{x_{21}}\\ \vdots \\ {\dot{e}}_{x_{n1}} \end{array}\right]=-\frac{1}{2}r\left[\begin{array}{c} x_{11}^{3}-y_{11}^{3}\\ x_{21}^{3}-y_{21}^{3}\\ \vdots \\ x_{n1}^{3}-y_{n1}^{3} \end{array}\right]+\frac{1}{2}\left(1+r\right)\left[\begin{array}{c} x_{11}^{2}-y_{11}^{2}\\ x_{21}^{2}-y_{21}^{2}\\ \vdots \\ x_{n1}^{2}-y_{n1}^{2} \end{array}\right]-\left[\begin{array}{c} e_{x_{11}}\\ e_{x_{21}}\\ \vdots \\ e_{x_{n1}} \end{array}\right]-\left[\begin{array}{c} e_{y_{n1}}\\ e_{y_{n1}}\\ \vdots \\ e_{y_{n1}} \end{array}\right]+\left[\begin{array}{c} \sum_{j=1}^{N}g_{1j}\frac{\left(x_{i1}-y_{i1}\right)}{2}\\ \sum_{j=1}^{N}g_{2j}\frac{\left(x_{i1}-y_{i1}\right)}{2}\\ \vdots \\ \sum_{j=1}^{N}g_{nj}\frac{\left(x_{i1}-y_{i1}\right)}{2} \end{array}\right]+\left[\begin{array}{c} u_{11}\\ u_{21}\\ \vdots \\ u_{n1} \end{array}\right],\\ \left[\begin{array}{c} {\dot{e}}_{y_{11}}\\ {\dot{e}}_{y_{21}}\\ \vdots \\ {\dot{e}}_{y_{n1}} \end{array}\right]=b\left[\begin{array}{c} e_{x_{11}}\\ e_{x_{21}}\\ \vdots \\ e_{x_{n1}} \end{array}\right]-c\left[\begin{array}{c} e_{y_{n1}}\\ e_{y_{n1}}\\ \vdots \\ e_{y_{n1}} \end{array}\right], \end{array}$$

where *u*_*i*1_=*u*_*x*_*i*1__ − *u*_*y*_*i*1__. Now, let us define the following terms for simplification:

(9) $$\begin{array}{c} e_{x_{1}}={\left[\begin{array}{cccc} e_{x_{11}} & e_{x_{21}} & \ldots & e_{x_{n1}} \end{array}\right]}^{T},\\ e_{y_{1}}={\left[\begin{array}{cccc} e_{y_{11}} & e_{y_{21}} & \ldots & e_{y_{n1}} \end{array}\right]}^{T},\\ c_{d}={\left[\begin{array}{cccc} x_{11}^{3}-y_{11}^{3} & x_{21}^{3}-y_{21}^{3} & \ldots & x_{n1}^{3}-y_{n1}^{3} \end{array}\right]}^{T},\\ s_{d}={\left[\begin{array}{cccc} x_{11}^{2}-y_{11}^{2} & x_{21}^{2}-y_{21}^{2} & \ldots & x_{n1}^{2}-y_{n1}^{2} \end{array}\right]}^{T},\\ G={\left(g_{ij}\right)}_{N\times N},\\ u={\left[\begin{array}{cccc} u_{11} & u_{21} & \ldots & u_{n1} \end{array}\right]}^{T}, \end{array}$$

where **e**_**x**_1__, **e**_**y**_1__, **c**_**d**_, **s**_**d**_, **u** ∈ *ℜ*^*Nx*1^, **G** ∈ *ℜ*^*NxN*^, and *T* represents the transpose operator. As a result, (8) can be written as follows:

(10) $$\begin{array}{c} {\dot{e}}_{x_{1}}=-\frac{1}{2}rc_{d}+\frac{1}{2}\left(1+r\right)s_{d}-e_{x_{1}}-e_{y_{1}}+Ge_{x_{1}}+u,\\ {\dot{e}}_{y_{1}}=be_{x_{1}}-ce_{y_{1}}. \end{array}$$

It can be concluded that the problem of synchronization is substituted with the synchronized error system (10) with the requirement to stabilize by using a suitable control input **u**. Synchronization can be achieved by designing the controller **u** such that for any initial conditions **e**_**x**_1__ and **e**_**y**_1__ converge to zero. This implies that the dynamics of the slave system (2/5) can converge to that of the drive system (1/4).

The article "Lag Synchronization of Noisy and Nonnoisy Multiple Neurobiological Coupled FitzHugh–Nagumo Networks with and without Delayed Coupling" was published in 2022. Journal: Comput Intell Neurosci.

Next, the Lyapunov stability and adaptive control theories are utilized to design a unique and simple control scheme that will guarantee the synchronization of the coupled FHN neurobiological without delay networks.

**Theorem 1 .**

Consider the nonnoisy/noisy multiple FHN neurobiological nondelayed networks described in equations (1) and (2) and (4) and (5) with the error dynamics described by equation (8). If the control laws in the error system described by equation (10) are designed as *u*_*i*1_={2**e**_**x**_1__(*g*_*i*1_+(*A*/*w*)sin(*wt*)+*b*_*i*1_+*c*_*i*1_) − 2**e**_**y**_1__(*g*_*i*2_ − (*A*/*w*)cos(*wt*) − *b*_*i*1_ − *c*_*i*1_)} then the synchronization of the nonnoisy/noisy multiple FHN coupled neurobiological non-delayed networks can be achieved.

**Proof**

The proof of this theorem and sufficient conditions that ensured the synchronization can be obtained using the theory of the Lyapunov stability. According to the theory of the Lyapunov stability, the stability of a system can be proved by choosing a positive definite function called as the Lyapunov function candidate *V*. In this study, it is chosen as follows:

(11) $$\begin{array}{c} V=\frac{1}{2}\left(e_{x_{1}}^{2}+e_{y_{1}}^{2}\right), \end{array}$$

d*v*/d*t* < 0 for all *t*.

It is easy to verify that the chosen candidate function *V* is a positive definite function. After taking the time derivative of (11), we obtain the following:

(12) $$\begin{array}{c} \dot{V}=e_{x_{1}}^{T}{\dot{e}}_{x_{1}}+e_{y_{1}}^{T}{\dot{e}}_{y_{1}}{\;}_{y_{1}}. \end{array}$$

Incorporating the synchronized error system (8) and the control laws into (12) yields the following:

(13) $$\begin{array}{c} \dot{V}=\left\{\begin{array}{c} e_{x_{1}}^{T}\left(\begin{array}{c} -\frac{1}{2}rc_{d}+\frac{1}{2}\left(1+r\right)s_{d}-e_{x_{1}}-e_{y_{1}}+2Ge_{x_{1}}+2e_{x_{1}}\left(g_{i1}+\left(\frac{A}{w}\right)\sin\left(wt\right)+b_{i1}+c_{i1}\right)\\ -2e_{y_{1}}\left(g_{i2}-\left(\frac{A}{w}\right)\cos\left(wt\right)-b_{i1}-c_{i1}\right) \end{array}\right)\\ +e_{y_{1}}^{T}\left(b_{i1}e_{x_{1}}-c_{i1}e_{y_{1}}\right) \end{array}\right\}, \end{array}$$

(14) $$\begin{array}{c} \dot{V}=\left(\begin{array}{c} -\frac{1}{2}re_{x_{1}}^{T}c_{d}+\frac{1}{2}\left(1+r\right)e_{x_{1}}^{T}s_{d}-e_{x_{1}}^{T}e_{x_{1}}-e_{x_{1}}^{T}e_{y_{1}}+2e_{x_{1}}^{T}Ge_{x_{1}}+2e_{x_{1}}^{T}e_{x_{1}}g_{i1}+\\ 2e_{x_{1}}^{T}e_{x_{1}}\left(\frac{A}{w}\right)\sin\left(wt\right)+2e_{x_{1}}^{T}e_{x_{1}}b_{i1}+2e_{x_{1}}^{T}e_{x_{1}}c_{i1}-2e_{x_{1}}^{T}e_{y_{1}}g_{i2}+2e_{x_{1}}^{T}e_{y_{1}}\left(\frac{A}{w}\right)\cos\left(wt\right)\\ +2e_{x_{1}}^{T}e_{y_{1}}b_{i1}+2e_{x_{1}}^{T}e_{y_{1}}c_{i1}+b_{i1}e_{y_{1}}^{T}e_{x_{1}}-c_{i1}e_{y_{1}}^{T}e_{y_{1}} \end{array}\right). \end{array}$$

Now,

(15) $$\begin{array}{c} e_{x_{1}}^{T}s_{d}=\left[\begin{array}{cccc} e_{x_{11}} & e_{x_{21}} & \ldots & e_{x_{n1}} \end{array}\right]\left[\begin{array}{c} \left(x_{11}+y_{11}\right)e_{x_{11}}\\ \left(x_{21}+y_{21}\right)e_{x_{21}}\\ \vdots \\ \left(x_{n1}+y_{n1}\right)e_{x_{n1}} \end{array}\right]\leq \left[\begin{array}{cccc} e_{x_{11}} & e_{x_{21}} & \ldots & e_{x_{n1}} \end{array}\right]\left[\begin{array}{c} \left(\left|x_{11}\right|+\left|y_{11}\right|\right)e_{x_{11}}\\ \left(\left|x_{21}\right|+\left|y_{21}\right|\right)e_{x_{21}}\\ \vdots \\ \left(\left|x_{n1}\right|+\left|y_{n1}\right|\right)e_{x_{n1}} \end{array}\right]. \end{array}$$

Moreover, it is known that neurons have bounded trajectories i.e., system (1) and (2) and (4) and (5) are bounded with some positive constant *q*_*x*_*i*__ and *q*_*y*_*i*__ satisfying |*x*_*i*1_| ≤ *q*_*x*_*i*__ and |*y*_*i*1_| ≤ *q*_*y*_*i*__, ∀*i*=1,2,3 …, *n*. Additionally, assuming that *q*_1_=max(*q*_*x*_*i*__+*q*_*y*_*i*__; *i*=1,2,3 …, *n*), (15) results into

(16) $$\begin{array}{c} e_{x_{1}}^{T}s_{d}\leq q_{1}e_{x_{1}}^{T}e_{x_{1}}. \end{array}$$

Correspondingly,

(17) $$\begin{array}{c} e_{x_{1}}^{T}c_{d}\leq q_{2}e_{x_{1}}^{T}e_{x_{1}}. \end{array}$$

Incorporating (16) and (17) into (14) gives

(18) $$\begin{array}{c} \dot{V}\leq -\left(\begin{array}{c} e_{x_{1}}^{T}e_{x_{1}}\left(\frac{1}{2}r-\frac{1}{2}\left(1+r\right)+I-2G-2g_{i1}-2\left(\frac{A}{w}\right)\sin\left(wt\right)-2b_{i1}-2c_{i1}\right)\\ +e_{x_{1}}^{T}e_{y_{1}}\left(I+2g_{i2}-2\left(\frac{A}{w}\right)\cos\left(wt\right)-2b_{i1}-2c_{i1}\right)\\ -b_{i1}e_{y_{1}}^{T}Ie_{x_{1}}+c_{i1}e_{y_{1}}^{T}Ie_{y_{1}} \end{array}\right). \end{array}$$

where **I** ∈ *ℜ*^*N*×*N*^, is the identity matrix,

(19) $$\begin{array}{c} \dot{V}\left(t\right)\leq -EPE^{T}, \end{array}$$

where $E=\left[\begin{array}{c} e_{x_{1}}\\ e_{y_{1}} \end{array}\right]$ and $P=\left[\begin{array}{cc} \left(\begin{array}{c} 1/2r-1/2\left(1+r\right)+I-2G-2g_{i1}\\ -2\left(A/w\right)\sin\left(wt\right)-2b_{i1}-2c_{i1} \end{array}\right) & \left(\begin{array}{c} I+2g_{i2}-2\left(A/w\right)\cos\left(wt\right)\\ -2b_{i1}-2c_{i1} \end{array}\right)\\ -b_{i1}I & c_{i1}I \end{array}\right]$.

The article "Lag Synchronization of Noisy and Nonnoisy Multiple Neurobiological Coupled FitzHugh–Nagumo Networks with and without Delayed Coupling" was published in 2022. Journal: Comput Intell Neurosci.

It can be concluded that the matrix **P** should be a positive definite to ensure the asymptotic stability of the synchronized error system (10) at the origin. The positive definiteness of **P** could be easily derived for considered networks of neurons (e.g., a network of five neurons) using the method of determinants, i.e., determinants of all leading principal minors have positive values [5]. Accordingly, the origin of the error system (10) is asymptotically stable. Consequently, these networks of n-identical neurobiological FHN neurons, under ionic gates disturbance, EES, and with and without external noise will achieve synchronization. This completes the proof.

### 2.2. FHN Multiple Delayed Neurobiological Networks

Multiple neurobiological noisy and nonnoisy FHN networks are modeled with delays in gap-junction dynamics.

#### 2.2.1. Multiple Delayed Neurobiological Nonnoisy FHN Networks

Let us consider nonnoisy multiple FHN neurobiological delayed networks composed of *n* neurons. Mathematically,

(20) $$\begin{array}{c} {\dot{x}}_{i1}=x_{i1}\left(x_{i1}-1\right)\left(1-r_{i1}x_{i1}\right)-x_{i2}+\sum_{j=1}^{n}g_{ij}x_{j1}\left(t-\tau_{1}\right)+I_{i1}+d_{i1}+u_{x_{i1}},\\ {\dot{x}}_{i2}=b_{i1}x_{i1}-c_{i1}x_{i2}\;i=1,2,3,\ldots ,n, \end{array}$$

(21) $$\begin{array}{c} {\dot{y}}_{i1}=y_{i1}\left(y_{i1}-1\right)\left(1-r_{i1}y_{i1}\right)-y_{i2}+\sum_{j=1}^{n}g_{ij}y_{j1}\left(t-\tau_{2}\right)+I_{i1}+d_{i1}+u_{y_{i1}},\\ {\dot{y}}_{i2}=b_{i1}y_{i1}-c_{i1}y_{i2}. \end{array}$$

#### 2.2.2. Multiple Delayed Neurobiological Noisy FHN Networks

Let us consider noisy multiple FHN neurobiological delayed networks composed of n neurons. Mathematically,

(22) $$\begin{array}{c} {\dot{x}}_{i1}=x_{i1}\left(x_{i1}-1\right)\left(1-r_{i1}x_{i1}\right)-x_{i2}+\sum_{j=1}^{n}g_{ij}x_{j1}\left(t-\tau_{1}\right)+I_{i1}+d_{i1}+\xi_{i1},\\ {\dot{x}}_{i2}=b_{i1}x_{i1}-c_{i1}x_{i2}\;i=1,2,3,\ldots ,n, \end{array}$$

(23) $$\begin{array}{c} {\dot{y}}_{i1}=y_{i1}\left(y_{i1}-1\right)\left(1-r_{i1}y_{i1}\right)-y_{i2}+\sum_{j=1}^{n}g_{ij}y_{j1}\left(t-\tau_{2}\right)+I_{i1}+d_{i1}+\xi_{i1}+u_{i1},\\ {\dot{y}}_{i2}=b_{i1}y_{i1}-c_{i1}y_{i2}. \end{array}$$

The article "Lag Synchronization of Noisy and Nonnoisy Multiple Neurobiological Coupled FitzHugh–Nagumo Networks with and without Delayed Coupling" was published in 2022. Journal: Comput Intell Neurosci.

#### 2.2.3. Nonlinear Control Design for Multiple Delayed Neurobiological FHN Networks

The error states of the neurobiological FHN systems formulated in equations (20–23) can be designed as follows:

(24) $$\begin{array}{c} e_{x_{i1}}^{\tau }=\frac{x_{i1}\left(t-\tau_{1}\right)-y_{i1}\left(t-\tau_{2}\right)}{2},\\ e_{y_{i1}}^{\tau }=\frac{x_{i2}\left(t-\tau_{1}\right)-y_{i2}\left(t-\tau_{2}\right)}{2}. \end{array}$$

Taking the derivative of the error system (17) with respect to time yields

(25) $$\begin{array}{c} \left[\begin{array}{c} {\dot{e}}_{x_{11}}^{\tau }\\ {\dot{e}}_{x_{21}}^{\tau }\\ \vdots \\ {\dot{e}}_{x_{n1}}^{\tau } \end{array}\right]=\left\{\begin{array}{c} -\frac{1}{2}r\left[\begin{array}{c} x_{11}^{3}\left(t-\tau_{1}\right)-y_{11}^{3}\left(t-\tau_{2}\right)\\ x_{21}^{3}\left(t-\tau_{1}\right)-y_{21}^{3}\left(t-\tau_{2}\right)\\ \vdots \\ x_{n1}^{3}\left(t-\tau_{1}\right)-y_{n1}^{3}\left(t-\tau_{2}\right) \end{array}\right]+\frac{1}{2}\left(1+r\right)\left[\begin{array}{c} x_{11}^{2}\left(t-\tau_{1}\right)-y_{11}^{2}\left(t-\tau_{2}\right)\\ x_{21}^{2}\left(t-\tau_{1}\right)-y_{21}^{2}\left(t-\tau_{2}\right)\\ \vdots \\ x_{n1}^{2}\left(t-\tau_{1}\right)-y_{n1}^{2}\left(t-\tau_{2}\right) \end{array}\right]-\left[\begin{array}{c} e_{x_{11}}^{\tau }\\ e_{x_{21}}^{\tau }\\ \vdots \\ e_{x_{n1}}^{\tau } \end{array}\right]-\left[\begin{array}{c} e_{y_{11}}^{\tau }\\ e_{y_{21}}^{\tau }\\ \vdots \\ e_{y_{n1}}^{\tau } \end{array}\right]\\ +\left[\begin{array}{c} \sum_{j=1}^{N}g_{1j}\frac{\left(x_{i1}\left(t-\tau_{1}\right)-y_{i1}\left(t-\tau_{2}\right)\right)}{2}\\ \sum_{j=1}^{N}g_{2j}\frac{\left(x_{i1}\left(t-\tau_{1}\right)-y_{i1}\left(t-\tau_{2}\right)\right)}{2}\\ \vdots \\ \sum_{j=1}^{N}g_{nj}\frac{\left(x_{i1}\left(t-\tau_{1}\right)-y_{i1}\left(t-\tau_{2}\right)\right)}{2} \end{array}\right]+\left[\begin{array}{c} u_{11}\\ u_{21}\\ \vdots \\ u_{n1} \end{array}\right] \end{array}\right\},\\ \left[\begin{array}{c} {\dot{e}}_{y_{11}}^{\tau }\\ {\dot{e}}_{y_{21}}^{\tau }\\ \vdots \\ {\dot{e}}_{y_{n1}}^{\tau } \end{array}\right]=b\left[\begin{array}{c} e_{x_{11}}^{\tau }\\ e_{x_{21}}^{\tau }\\ \vdots \\ e_{x_{n1}}^{\tau } \end{array}\right]-c\left[\begin{array}{c} e_{y_{11}}^{\tau }\\ e_{y_{21}}^{\tau }\\ \vdots \\ e_{y_{n1}}^{\tau } \end{array}\right], \end{array}$$

where *u*_*i*1_=*u*_*x*_*i*1__ − *u*_*y*_*i*1__. Now, let us define the following terms for simplification,

(26) $$\begin{array}{c} e_{x_{1}}^{\tau }={\left[\begin{array}{cccc} e_{x_{11}}^{\tau } & e_{x_{21}}^{\tau } & \ldots & e_{x_{n1}}^{\tau } \end{array}\right]}^{T},\\ e_{y_{1}}^{\tau }={\left[\begin{array}{cccc} e_{y_{11}}^{\tau } & e_{y_{21}}^{\tau } & \ldots & e_{y_{n1}}^{\tau } \end{array}\right]}^{T},\\ c_{d}^{\tau }={\left[\begin{array}{cccc} x_{11}^{3}\left(t-\tau_{1}\right)-y_{11}^{3}\left(t-\tau_{2}\right) & x_{21}^{3}\left(t-\tau_{1}\right)-y_{21}^{3}\left(t-\tau_{2}\right) & \ldots & x_{n1}^{3}\left(t-\tau_{1}\right)-y_{n1}^{3}\left(t-\tau_{2}\right) \end{array}\right]}^{T},\\ s_{d}^{\tau }={\left[\begin{array}{cccc} x_{11}^{2}\left(t-\tau_{1}\right)-y_{11}^{2}\left(t-\tau_{2}\right) & x_{21}^{2}\left(t-\tau_{1}\right)-y_{21}^{2}\left(t-\tau_{2}\right) & \ldots & x_{n1}^{2}\left(t-\tau_{1}\right)-y_{n1}^{2}\left(t-\tau_{2}\right) \end{array}\right]}^{T},\\ G={\left(g_{ij}\right)}_{N\times N},\\ u={\left[\begin{array}{cccc} u_{11} & u_{21} & \ldots & u_{n1} \end{array}\right]}^{T}, \end{array}$$

where **e**_**x**_1__^*τ*^, **e**_**y**_1__^*τ*^, **c**_**d**_^*τ*^, **s**_**d**_^*τ*^, **u** ∈ *ℜ*^*N*×1^, **G** ∈ *ℜ*^*N*×*N*^ and *T* represents the transpose operator. As a result, (25) can be written as follows:

(27) $$\begin{array}{c} {\dot{e}}_{x_{1}}^{\tau }=-\frac{1}{2}rc_{d}^{\tau }+\frac{1}{2}\left(1+r\right)s_{d}^{\tau }-e_{x_{1}}^{\tau }-e_{y_{1}}^{\tau }+Ge_{x_{1}}^{\tau }+u,\\ {\dot{e}}_{y_{1}}^{\tau }=be_{x_{1}}^{\tau }-ce_{y_{1}}^{\tau }. \end{array}$$

It can be concluded that the problem of synchronization is substituted with the synchronized error system (27) with the requirement to stabilize by using a suitable control input **u**. Synchronization can be achieved by designing the controller **u** such that for any initial conditions **e**_**x**_1__^*τ*^ and **e**_**y**_1__^*τ*^ converge to zero. This implies that the dynamics of the slave system (20/22) can converge to that of the drive system (19/21).

The article "Lag Synchronization of Noisy and Nonnoisy Multiple Neurobiological Coupled FitzHugh–Nagumo Networks with and without Delayed Coupling" was published in 2022. Journal: Comput Intell Neurosci.

**Theorem 2 .**

Consider the nonnoisy/noisy multiple FHN neurobiological delayed systems as described in equations (20–23) with the error dynamics described by equation (25). If the controllers defined in equation (27) are designed as *u*_*i*1_={−*g*_*i*1_(*b*_*i*1_ − *c*_*i*1_)**e**_**x**_1__^*τ*^ − (*b*_*i*1_ − *c*_*i*1_)**e**_**y**_1__^*τ*^}, then the synchronization of the nonnoisy/noisy multiple FHN neurobiological delayed networks presented in equations (20–23) can be achieved.

**Proof**

The Lyapunov function candidate *V* is chosen as follows:

(28) $$\begin{array}{c} V=\frac{1}{2}\left(e_{x_{1}}^{\tau 2}+e_{y_{1}}^{\tau 2}\right), \end{array}$$

d*v*/d*t* < 0 for all *t*.

It is easy to verify that the chosen candidate function *V* is a positive definite function. After taking the time derivative of (27), we obtain the following:

(29) $$\begin{array}{c} \dot{V}=e_{x_{1}}^{\tau T}{\dot{e}}_{x_{1}}^{\tau }+e_{y_{1}}^{\tau T}{\dot{e}}_{y_{1}}^{\tau }. \end{array}$$

Incorporating the synchronized error system (25) and the control laws into (29) yields the following:

(30) $$\begin{array}{c} \dot{V}=\left\{\begin{array}{c} e_{x_{1}}^{\tau Τ}\left(-\frac{1}{2}rc_{d}^{\tau }+\frac{1}{2}\left(1+r\right)s_{d}^{\tau }-e_{x_{1}}^{\tau }-e_{y_{1}}^{\tau }+Ge_{x_{1}}^{\tau }-g_{i1}\left(b_{i1}-c_{i1}\right)e_{x_{1}}^{\tau }-\left(b_{i1}-c_{i1}\right)e_{y_{1}}^{\tau }\right)\\ +e_{x_{1}}^{\tau Τ}\left(b_{i1}e_{x_{1}}^{\tau }-c_{i1}e_{y_{1}}^{\tau }\right) \end{array}\right\}, \end{array}$$

(31) $$\begin{array}{c} \dot{V}=-\left\{\begin{array}{c} \frac{1}{2}re_{x_{1}}^{\tau Τ}c_{d}^{\tau }-\frac{1}{2}\left(1+r\right)e_{x_{1}}^{\tau Τ}s_{d}^{\tau }+e_{x_{1}}^{\tau Τ}e_{x_{1}}^{\tau }+e_{x_{1}}^{\tau Τ}e_{y_{1}}^{\tau }-Ge_{x_{1}}^{\tau Τ}e_{x_{1}}^{\tau }+g_{i1}\left(b_{i1}-c_{i1}\right)e_{x_{1}}^{\tau Τ}e_{x_{1}}^{\tau }\\ +\left(b_{i1}-c_{i1}\right)e_{x_{1}}^{\tau Τ}e_{y_{1}}^{\tau }-b_{i1}e_{y_{1}}^{\tau Τ}e_{x_{1}}^{\tau }+c_{i1}e_{y_{1}}^{Τ\tau }e_{y_{1}}^{\tau } \end{array}\right\},\dot{V}=-\left\{\begin{array}{c} \frac{1}{2}re_{x_{1}}^{\tau Τ}c_{d}^{\tau }-\frac{1}{2}\left(1+r\right)e_{x_{1}}^{\tau Τ}s_{d}^{\tau }+e_{x_{1}}^{\tau Τ}e_{x_{1}}^{\tau }+e_{x_{1}}^{\tau Τ}e_{y_{1}}^{\tau }-Ge_{x_{1}}^{\tau Τ}e_{x_{1}}^{\tau }+g_{i1}\left(b_{i1}-c_{i1}\right)e_{x_{1}}^{\tau Τ}e_{x_{1}}^{\tau }\\ +\left(b_{i1}-c_{i1}\right)e_{x_{1}}^{\tau Τ}e_{y_{1}}^{\tau }-b_{i1}e_{y_{1}}^{\tau Τ}e_{x_{1}}^{\tau }+c_{i1}e_{y_{1}}^{\tau Τ}e_{y_{1}}^{\tau } \end{array}\right\}, \end{array}$$

(32) $$\begin{array}{c} \text{Now }e_{x_{1}}^{\tau Τ}s_{d}^{\tau }=\left\{\begin{array}{c} \left[\begin{array}{cccc} e_{x_{11}}^{\tau } & e_{x_{21}}^{\tau } & \ldots & e_{x_{n1}}^{\tau } \end{array}\right]\left[\begin{array}{c} \left(x_{11}\left(t-\tau_{1}\right)+y_{11}\left(t-\tau_{2}\right)\right)e_{x_{11}}^{\tau }\\ \left(x_{21}\left(t-\tau_{1}\right)+y_{21}\left(t-\tau_{2}\right)\right)e_{x_{21}}^{\tau }\\ \vdots \\ \left(x_{n1}\left(t-\tau_{1}\right)+y_{n1}\left(t-\tau_{2}\right)\right)e_{x_{n1}}^{\tau } \end{array}\right]\leq \\ \left[\begin{array}{cccc} e_{x_{11}}^{\tau } & e_{x_{21}}^{\tau } & \ldots & e_{x_{n1}}^{\tau } \end{array}\right]\left[\begin{array}{c} \left(\left|x_{11}\left(t-\tau_{1}\right)\right|+\left|y_{11}\left(t-\tau_{2}\right)\right|\right)e_{x_{11}}^{\tau }\\ \left(\left|x_{21}\left(t-\tau_{1}\right)\right|+\left|y_{21}\left(t-\tau_{2}\right)\right|\right)e_{x_{21}}^{\tau }\\ \vdots \\ \left(\left|x_{n1}\left(t-\tau_{1}\right)\right|+\left|y_{n1}\left(t-\tau_{2}\right)\right|\right)e_{x_{n1}}^{\tau } \end{array}\right] \end{array}\right\}. \end{array}$$

Moreover, it is known that neurons have bounded trajectories, i.e., the system (20–23) are bounded with some positive constant *q*_*x*_*i*__ and *q*_*y*_*i*__ satisfying |*x*_*i*1_| ≤ *q*_*x*_*i*__ and |*y*_*i*1_| ≤ *q*_*y*_*i*__, ∀*i*=1,2,3 …, *n*. Additionally, assuming that *q*_1_=max(*q*_*x*_*i*__+*q*_*y*_*i*__; *i*=1,2,3 …, *n*), (32) results into the following:

(33) $$\begin{array}{c} e_{x_{1}}^{\tau T}s_{d}^{\tau }\leq q_{1}e_{y_{1}}^{\tau T}e_{x_{1}}^{\tau }. \end{array}$$

Correspondingly,

(34) $$\begin{array}{c} e_{y_{1}}^{\tau T}c_{d}^{\tau }\leq q_{2}e_{x_{1}}^{\tau T}e_{x_{1}}^{\tau }. \end{array}$$

Incorporating (33) and (34) into (31) gives

(35) $$\begin{array}{c} \dot{V}\leq -\left\{\begin{array}{c} e_{x_{1}}^{\tau T}\left(\frac{1}{2}rq_{2}-\frac{1}{2}\left(1+r\right)q_{1}+I-G+g_{i1}b_{i1}-g_{i1}c_{i1}\right)e_{x_{1}}^{\tau }+e_{x_{1}}^{\tau T}\left(I+b_{i1}-c_{i1}\right)e_{y_{1}}^{\tau }\\ -b_{i1}e_{y_{1}}^{\tau T}Ie_{x_{1}}^{\tau }+c_{i1}e_{Y_{1}}^{\tau T}Ie_{y_{1}}^{\tau } \end{array}\right\}, \end{array}$$

where **I** ∈ *ℜ*^*N*×*N*^ is the identity matrix.

(36) $$\begin{array}{c} \dot{V}\left(t\right)\leq -EPE^{T}, \end{array}$$

where $E=\left[\begin{array}{c} e_{x_{1}}\\ e_{y_{1}} \end{array}\right]$ and $P=\left[\begin{array}{cc} 1/2rq_{2}-1/2\left(1+r\right)q_{1}+I-G+g_{i1}b_{i1}-g_{i1}c_{i1} & I+b_{i1}-c_{i1}\\ -b_{i1}I & c_{i1}I \end{array}\right]$.

The article "Lag Synchronization of Noisy and Nonnoisy Multiple Neurobiological Coupled FitzHugh–Nagumo Networks with and without Delayed Coupling" was published in 2022. Journal: Comput Intell Neurosci.

It can be concluded that the matrix **P** should be a positive definite to ensure the asymptotic stability of the synchronized error system (26) at the origin. The positive definiteness of **P** could be easily derived for considered networks of neurons (e.g., a network of five neurons) using the method of determinants, i.e., determinants of all leading principal minors have positive values [5]. Accordingly, the origin of the error system (26) is asymptotically stable. Consequently, these networks of n-identical delayed neurobiological FHN neural network composed of n neurons, under ionic gates disturbance, EES, and with and without external noise will achieve synchronization. This completes the proof.

## 3. Numerical Results

In this section, the results of the numerical simulations are discussed to analyze and validate the efficacy of the designed control laws for the synchronization of noisy and nonnoisy multiple neurobiological FHN networks with and without delayed gap junctions. To perform this, we considered five neurons of two noisy and nonnoisy multiple neurobiological FHN networks with and without delay gap-junctions and external noise. The parameter values used in this study are *r*_11_ = 10, *r*_21_ = 10.2, *r*_31_ = 10.4, *r*_41_ = 10.6, *r*_51_ = 10.8, *b*_11_ = 1, *b*_21_ = 1.001, *b*_31_ = 1.002, *b*_41_ = 1.003, *b*_51_ = 1.004, *c*_11_ = 0.001, *c*_21_ = 0.002, *c*_31_ = 0.003, *c*_41_ = 0.004, *c*_51_ = 0.005, *d*_11_ = 0.001 sin(0.2 × *t*), *d*_21_ = 0.002 sin(0.2 × *t*), *d*_31_ = 0.003 sin(0.2 × *t*), *d*_41_ = 0.004 sin(0.2 × *t*), *d*_51_ = 0.005 sin(0.2 × *t*), *A* = 0.1, *f* = 0.129, *ω* = 2*πf* and initial conditions are *x*_11_(0) = 0, *y*_11_(0) = 0, *x*_12_(0) = 0.1, *y*_12_(0) = 0.1, *x*_21_(0) = 0.05, *y*_21_(0) = 0.05, *x*_22_(0) = 0.2, *y*_22_(0) = 0.2, *x*_31_(0) = 0.05, *y*_31_(0) = 0.05, *x*_32_(0) = 0.2, *y*_22_(0) = 0.2, *x*_41_(0) = 0, *y*_41_(0) = 0, *x*_42_(0) = 0.1, *y*_42_(0) = 0.1, *x*_51_(0) = 0.05, *y*_51_(0) = 0.05, *x*_52_(0) = 0.2, and *y*_52_(0) = 0.2. The values of the gap junctions are listed in the matrix **G**

(37) $$\begin{array}{c} G=\left[\begin{array}{ccccc} -1.0735\times 10^{-03} & 3\text{.}6412\times 10^{-04} & 4.0396\times 10^{-04} & 2.064\times 10^{-05} & 2\text{.}8481\times 10^{-04}\\ 3\text{.}6412\times 10^{-04} & -1\text{.}5070\times 10^{-03} & 8\text{.}3269\times 10^{-04} & 1\text{.}6223\times 10^{-04} & 1\text{.}4797\times 10^{-04}\\ 4.0396\times 10^{-04} & 8\text{.}3269\times 10^{-04} & -2\text{.}2451\times 10^{-03} & 8\text{.}1832\times 10^{-04} & 1\text{.}9013\times 10^{-04}\\ 2.064\times 10^{-05} & 1\text{.}6223\times 10^{-04} & 8\text{.}1832\times 10^{-04} & -1\text{.}6371\times 10^{-03} & 6\text{.}3596\times 10^{-04}\\ 2\text{.}8481\times 10^{-04} & 1\text{.}4797\times 10^{-04} & 1\text{.}9013\times 10^{-04} & 6\text{.}3596\times 10^{-04} & -1\text{.}2589\times 10^{-03} \end{array}\right]. \end{array}$$

Figures 2(a)–2(e) and 3(a)–3(e) illustrate the errors in temporal dynamics with (red lines) and without (blue lines) proposed control laws for nonnoisy coupled FHN networks without delay for membrane potential states and recovery variables states, respectively. The nonconverging behavior observed through spiked errors for both membrane potential states and recovery states of each network revealed the unsynchronized activities of the networks (Figures 2(a)–2(e) and 3(a)–3(e), blue lines). We used the strategy of controller switch off and on for critically analyzing and evaluating the performance of the proposed control scheme. As shown in Figures 2(a)–2(e) and 3(a)–3(e) (red lines), the proposed controller was not applied until *t* = 150 and the temporal dynamics of the neurons is highly abrupt, but all the errors converged to zero, proving synchronization between both states of all neurons in both networks, as soon as the designed control laws are activated, showing the efficacy of the proposed scheme.

The article "Lag Synchronization of Noisy and Nonnoisy Multiple Neurobiological Coupled FitzHugh–Nagumo Networks with and without Delayed Coupling" was published in 2022. Journal: Comput Intell Neurosci.

Furthermore, the unsynchronized activities of the networks could also be observed through the abrupt behavior of the phase plane diagrams for both states as shown in Figures 4(a)–4(e) and 5(a)–5(e). In addition, the straight lines in phase plane diagrams (Figures 4(a)–4(e) and 5(a)–5(e), red lines) after the application of designed control laws indicate that both membrane potential states and recovery variable states of each neuron in both networks have synchronized activities.

Figures 6(a)–6(e) and 7(a)–7(e) illustrate the errors in temporal dynamics with (red lines) and without (blue lines) proposed control laws for noisy multiple FHN without delayed coupling for membrane potential states and recovery variables states, respectively. The nonconverging behavior observed through spiked errors for both membrane potential states and recovery states of each network revealed the unsynchronized activities of the networks (Figures 6(a)–6(e) and 7(a)–7(e), blue lines). We used the strategy of controller switch off and on for critically analyzing and evaluating the performance of the proposed control scheme. As shown in Figures 6(a)–6(e) and 7(a)–7(e)) (red lines), the proposed controller was not applied until *t* = 150 and the temporal dynamics of the neurons is highly abrupt, but all the errors converged to zero, proving synchronization between both states of all neurons in both networks, as soon as the designed control laws are activated, showing the efficacy of the proposed scheme. Furthermore, the unsynchronized activities of the network could also be observed through the abrupt behavior of the phase plane diagrams for both states as shown in Figures 8(a)–8(e) and 9(a)–9(e). In addition, the straight lines in phase plane diagrams (Figures 8(a)–8(e) and 9(a)–9(e), red lines) after the application of the designed control laws indicate that both membrane potential states and recovery variable states of each neuron in both networks have synchronized activities.

Figures 10(a)–10(e) and 11(a)–11(e) illustrate the errors in temporal dynamics with (red lines) and without (blue lines) proposed control laws for nonnoisy multiple FHN with delayed coupling for membrane potential states and recovery variables states, respectively. The nonconverging behavior observed through spiked errors for both membrane potential states and recovery states of each network revealed the unsynchronized activities of the networks (Figures 10(a)–10(e) and 11(a)–11(e), blue lines). We used the strategy of controller switches off and on for critically analyzing and evaluating the performance of the proposed control scheme. As shown in Figures 10(a)–10(e) and 11(a)–11(e) (red lines), the proposed controller was not applied until *t* = 110 and the temporal dynamics of the neurons is highly abrupt, but all the errors converged to zero, proving synchronization between both states of all neurons in both networks, as soon as the designed control laws are activated, showing the efficacy of the proposed scheme. Furthermore, the unsynchronized activities of the network could also be observed through the abrupt behavior of the phase plane diagrams for both states as shown in Figures 12(a)–12(e) and 13(a)–13(e). In addition, the straight lines in phase plane diagrams (Figures 12(a)–12(e) and 13(a)–13(e), red lines) after the application of designed control laws indicate that both membrane potential states and recovery variable states of each neuron in both networks have synchronized activities.

The article "Lag Synchronization of Noisy and Nonnoisy Multiple Neurobiological Coupled FitzHugh–Nagumo Networks with and without Delayed Coupling" was published in 2022. Journal: Comput Intell Neurosci.

Figures 14(a)–14(e) and 15(a)–15(e) illustrate the errors in temporal dynamics with (red lines) and without (blue lines) proposed control laws for noisy multiple FHN networks with delayed coupling for membrane potential states and recovery variables states, respectively. The nonconverging behavior observed through spiked errors for both membrane potential states and recovery states of each network revealed the unsynchronized activities of the networks (Figures 14(a)–14(e) and 15(a)–15(e), blue lines). We used the strategy of controller switch off and on for critically analyzing and evaluating the performance of the proposed control scheme. As shown in Figures 14(a)–14(e) and 15(a)–15(e) (red lines), the proposed controller was not applied until *t* = 110 and the temporal dynamics of the neurons is highly abrupt, but all the errors converged to zero, proving synchronization between both states of all neurons in both networks, as soon as the designed control laws are activated, showing the efficacy of the proposed scheme. Furthermore, the unsynchronized activities of the network could also be observed through the abrupt behavior of the phase plane diagrams for both states as shown in Figures 16(a)–16(e) and 17(a)–17(e) (blue lines). In addition, the straight lines in phase plane diagrams (Figures 16(a)–16(e) and 17(a)–17(e)), red lines) after the application of designed control laws indicate that both membrane potential states and recovery variable states of each neuron in both networks have synchronized activities.

## 4. Conclusion

This paper presents the design of different control schemes for the synchronization of noisy and nonnoisy multiple neurobiological FHN networks with and without delay coupling. Variable parameters have been used for each state of both FHN networks. The proposed control laws for both networks are different and unique to achieve synchronization. The robust adaptive control theory was utilized to propose robust and different adaptive control strategies to investigate the synchronization problem of the noisy and nonnoisy multiple neurobiological FHN networks with and without delay coupling. Control laws are designed to stabilize the error dynamics without direct cancelation and to synchronize all the states of both FHN neurobiological networks. Sufficient conditions for achieving synchronization in the multiple noisy and nonnoisy neurobiological networks were derived analytically using the Lyapunov stability theory. The results of numerical simulations demonstrated the efficacy of the designed control schemes. The most important contributions of this research consist of (i) examining the nondelayed multiple coupled FHN neurobiological networks under the conditions of external noise (with and without), different delayed gap-junctions, and external disturbance, (ii) examining the delayed multiple coupled FHN neurobiological networks under the conditions of external noise (with and without), different delayed gap-junctions and external disturbance, (iii) the development of novel and diverse control laws under the conditions of external noise (with and without) for both multiple FHN neurobiological delayed and nondelayed networks, and (iv) achieving the synchronization of multiple FHN neurobiological networks membrane states and recovery variables states for drive and slave networks using the proposed control schemes.

The article "Lag Synchronization of Noisy and Nonnoisy Multiple Neurobiological Coupled FitzHugh–Nagumo Networks with and without Delayed Coupling" was published in 2022. Journal: Comput Intell Neurosci.

## Figures and Tables

**Figure 1:** Schematic diagram showing a general configuration of coupled neurobiological FitzHugh–Nagumo (FHN).

**Figure 2:** Synchronization error dynamics between membrane potential states of nonnoisy multiple FHN neurobiological networks (redline: with control and blue line: without control). (a) Error dynamics *e*_*x*_11__=*x*_11_ − *y*_11_/2. (b) Error dynamics *e*_*x*_21__=*x*_21_ − *y*_21_/2. (c) Error dynamics *e*_*x*_31__=*x*_31_ − *y*_31_/2. (d) Error dynamics *e*_*x*_41__=*x*_41_ − *y*_41_/2. (e) Error dynamics *e*_*x*_51__=*x*_51_ − *y*_51_/2.

**Figure 3:** Synchronization error dynamics between recovery states of nonnoisy multiple FHN neurobiological networks (redline: with control and blue line: without control). (a) Error dynamics *e*_*y*_11__=*x*_12_ − *y*_12_/2 when *b*_11_=1, *c*_11_=0.001. (b) Error dynamics *e*_*y*_21__=*x*_22_ − *y*_22_/2. (c) Error dynamics *e*_*y*_31__=*x*_32_ − *y*_32_/2. (d) Error dynamics *e*_*y*_41__=*x*_42_ − *y*_42_/2. (e) Error dynamics *e*_*y*_51__=*x*_52_ − *y*_52_/2.

**Figure 4:** Synchronization analysis between membrane potential states of nonnoisy multiple FHN neurobiological networks (redline: with control and blue line: without control). (a) Phase plane *x*_11_ − *y*_11_. (b) Phase plane *x*_21_ − *y*_21_. (c) Phase plane *x*_31_ − *y*_31_. (d) Phase plane *x*_41_ − *y*_41_. (e) Phase plane *x*_51_ − *y*_51_.

The article "Lag Synchronization of Noisy and Nonnoisy Multiple Neurobiological Coupled FitzHugh–Nagumo Networks with and without Delayed Coupling" was published in 2022. Journal: Comput Intell Neurosci.

**Figure 5:** Synchronization analysis of the recovery variable states of nonnoisy multiple FHN neurobiological networks (redline: with control and blue line: without control). (a) Phase plane *x*_12_ − *y*_12_. (b) Phase plane *x*_22_ − *y*_22_. (c) Phase plane *x*_32_ − *y*_32_. (d) Phase plane *x*_42_ − *y*_42_. (e) Phase plane *x*_52_ − *y*_52_.

**Figure 6:** Synchronization error dynamics between membrane potential states of noisy multiple FHN neurobiological networks (redline: with control and blue line: without control). (a) Error dynamics *e*_*x*_11__=*x*_11_ − *y*_11_/2. (b) Error dynamics *e*_*x*_21__=*x*_21_ − *y*_21_/2. (c) Error dynamics *e*_*x*_31__=*x*_31_ − *y*_31_/2. (d) Error dynamics *e*_*x*_41__=*x*_41_ − *y*_41_/2. (e) Error dynamics *e*_*x*_51__=*x*_51_ − *y*_51_/2.

**Figure 7:** Synchronization error dynamics between recovery variable states of noisy multiple FHN neurobiological networks (redline: with control and blue line: without control). (a) Error dynamics *e*_*y*_11__=*x*_12_ − *y*_12_/2. (b) Error dynamics *e*_*y*_21__=*x*_22_ − *y*_22_/2. (c) Error dynamics *e*_*y*_31__=*x*_32_ − *y*_32_/2. (d) Error dynamics *e*_*y*_41__=*x*_42_ − *y*_42_/2. (e) Error dynamics *e*_*y*_51__=*x*_52_ − *y*_52_/2.

**Figure 8:** Synchronization analysis between membrane potential states of noisy multiple FHN neurobiological networks (redline: with control and blue line: without control). (a) Phase plane *x*_11_ − *y*_11_. (b) Phase plane *x*_21_ − *y*_21_. (c) Phase plane *x*_31_ − *y*_31_. (d) Phase plane *x*_41_ − *y*_41_. (e) Phase plane *x*_51_ − *y*_51_.

**Figure 9:** Synchronization analysis of the recovery variable states of noisy multiple FHN neurobiological networks (redline: with control and blue line: without control). (a) Phase plane *x*_12_ − *y*_12_. (b) Phase plane *x*_22_ − *y*_22_. (c) Phase plane *x*_32_ − *y*_32_. (d) Phase plane *x*_42_ − *y*_42_. (e) Phase plane *x*_52_ − *y*_52_.

**Figure 10:** Synchronization error dynamics between membrane potential states of nonnoisy multiple FHN neurobiological delayed networks (redline: with control and blue line: without control). (a) Error dynamics *e*_*x*_11__=*x*_11_ − *y*_11_/2. (b) Error dynamics *e*_*x*_21__=*x*_21_ − *y*_21_/2. (c) Error dynamics *e*_*x*_31__=*x*_31_ − *y*_31_/2. (d) Error dynamics *e*_*x*_41__=*x*_41_ − *y*_41_/2. (e) Error dynamics *e*_*x*_51__=*x*_51_ − *y*_51_/2.

**Figure 11:** Synchronization error dynamics between recovery variable states of nonnoisy multiple FHN neurobiological delayed networks (redline: with control and blue line: without control). (a) Error dynamics *e*_*y*_11__=*x*_12_ − *y*_12_/2. (b) Error dynamics *e*_*y*_21__=*x*_22_ − *y*_22_/2. (c) Error dynamics *e*_*y*_31__=*x*_32_ − *y*_32_/2. (d) Error dynamics *e*_*y*_41__=*x*_42_ − *y*_42_/2. (e) Error dynamics *e*_*y*_51__=*x*_52_ − *y*_52_/2.

The article "Lag Synchronization of Noisy and Nonnoisy Multiple Neurobiological Coupled FitzHugh–Nagumo Networks with and without Delayed Coupling" was published in 2022. Journal: Comput Intell Neurosci.

**Figure 12:** Synchronization analysis between membrane potential states of nonnoisy multiple FHN neurobiological delayed networks (redline: with control and blue line: without control). (a) Phase plane *x*_11_ − *y*_11_. (b) Phase plane *x*_21_ − *y*_21_. (c) Phase plane *x*_31_ − *y*_31_. (d) Phase plane *x*_41_ − *y*_41_. (e) Phase plane *x*_51_ − *y*_51_.

**Figure 13:** Synchronization analysis of the recovery variable states of nonnoisy multiple FHN neurobiological delayed networks (redline: with control and blue line: without control). (a) Phase plane *x*_12_ − *y*_12_. (b) Phase plane *x*_22_ − *y*_22_. (c) Phase plane *x*_32_ − *y*_32_. (d) Phase plane *x*_42_ − *y*_42_. (e) Phase plane *x*_52_ − *y*_52_.

**Figure 14:** Synchronization error dynamics between membrane potential states of noisy multiple FHN neurobiological delayed networks (redline: with control and blue line: without control). (a) Error dynamics *e*_*x*_11__=*x*_11_ − *y*_11_/2. (b) Error dynamics *e*_*x*_21__=*x*_21_ − *y*_21_/2. (c) Error dynamics *e*_*x*_31__=*x*_31_ − *y*_31_/2. (d) Error dynamics *e*_*x*_41__=*x*_41_ − *y*_41_/2. (e) Error dynamics *e*_*x*_51__=*x*_51_ − *y*_51_/2.

**Figure 15:** Synchronization error dynamics between recovery variable states of noisy multiple FHN neurobiological delayed networks (redline: with control and blue line: without control). (a) Error dynamics *e*_*y*_11__=*x*_12_ − *y*_12_/2. (b) Error dynamics *e*_*y*_21__=*x*_22_ − *y*_22_/2. (c) Error dynamics *e*_*y*_31__=*x*_32_ − *y*_32_/2. (d) Error dynamics *e*_*y*_41__=*x*_42_ − *y*_42_/2. (e) Error dynamics *e*_*y*_51__=*x*_52_ − *y*_52_/2.

**Figure 16:** Synchronization analysis between membrane potential states of noisy multiple FHN neurobiological delayed networks (redline: with control and blue line: without control). (a) Phase plane *x*_11_ − *y*_11_ (b) Phase plane *x*_21_ − *y*_21_. (c) Phase plane *x*_31_ − *y*_31_. (d) Phase plane *x*_41_ − *y*_41_. (e) Phase plane *x*_51_ − *y*_51_.

**Figure 17:** Synchronization analysis of the recovery variable states of noisy multiple FHN neurobiological delayed networks (redline: with control and blue line: without control). (a) Phase plane *x*_12_ − *y*_12_. (b) Phase plane *x*_22_ − *y*_22_. (c) Phase plane *x*_32_ − *y*_32_. (d) Phase plane *x*_42_ − *y*_42_. (e) Phase plane *x*_52_ − *y*_52_.

The article "Lag Synchronization of Noisy and Nonnoisy Multiple Neurobiological Coupled FitzHugh–Nagumo Networks with and without Delayed Coupling" was published in 2022. Journal: Comput Intell Neurosci.

## Data Availability

No data have been used.
